# Analysis of the Key Factors of Ecological Environment Protection in the National Economic Sustainable Development Goals

**DOI:** 10.1155/2022/3593587

**Published:** 2022-08-13

**Authors:** Haiwen Long

**Affiliations:** Business School, Yuxi Normal University, Yuxi 653100, China

## Abstract

Urbanization helps people to create comfortable and convenient living conditions and meets the needs of people survival, enjoyment, and development. At the same time, the surge in population has also caused great disturbance and damage to the urban natural environment. Humans continue to utilize and transform nature by increasing the absolute surface area of the natural environment, but at the same time, rapid population growth and scarcity of resources exacerbate the absurd development and utilization of resources, leading to ecological destruction. The development of green plants, animals, and other creatures is hindered, and the imbalance of urban ecology aggravates the contradiction between man and the ecological environment. Based on this, the paper first expounds on the theoretical framework of sustainable economic development, draws the analysis of the elements of sustainable economic development, and then studies the coupling relationship model between economic development and ecological environmental protection as an example of the regional economy. GM (1.1) principle was used to test the practicability of the model and found that the model is very accurate in predicting the coordinated development between economic development and ecological environmental protection. It provides a comprehensive index of the sustainable capacity of the ecological environment in urban areas, analyses the indicators of Leshan City, and draws a conclusion: the main factors affecting the sustainable development of Leshan's ecological environment are the economic environment and the natural environment; it is necessary to further adjust the industrial structure. In order to maintain sustained and stable economic development, it is very important to strengthen urban environmental protection, develop circular economy, and continuously improve the level of ecologically sustainable development.

## 1. Introduction

Researching and improving the ecological environment of arid areas in western China is of great significance to the implementation of national strategies and policies to accelerate the development of this area. The purpose of this project is to determine the dynamic carrying capacity and ecological water demand of arid areas in western China. At the same time, an ecological environment evolution model and an ecological environment information system have been established [1]. In an ecological environment, after inputting the reflective properties of the lower surface, the terrestrial solar radiation spectral flux on the clear sky level at any time of year, geographic location, and altitude can be calculated. The comparison of the measured values is consistent [2]. The Zoige Plateau has been showing signs of swamp degradation since the 1960s. Forty years later, the ecological environment has deteriorated, and swamp degradation has become increasingly serious. Compared with natural factors, the disturbance of human activities is the main reason for the deterioration of the ecological environment and swamp degradation [3]. Land consolidation is a process of rebuilding the ecological environment system, which has an impact on regional environmental factors and ecological processes. This paper proposes three factors that affect the regional ecological environment in the process of land consolidation, and analyses the impact of these factors on the regional ecological environment [4]. With the rapid development of the economy, the degree of people's exploitation of natural resources is increasing. Under the combined action of natural and human factors, the hydrological properties of wetlands have undergone tremendous changes. Therefore, the author takes Baiyangdian wetland as an example to study sustainable development strategies in order to achieve the harmonious development of ecology, society, and economy [5]. Official estimates of the cost of traffic accidents in 1990 or later, compiled from readily available information for 12 countries, have a segmental impact on national economies, and estimates of gross national product are taken from OECD publications [6]. In Ireland, where a recent study assessed the national and regional economic value of the maritime sector, the input-output approach could examine the linkages and impact of Irish maritime revenues on the national economy. This analysis shows that Ireland's economic support mostly depends on seafood [7]. Ghana's minerals and mining sector has seen a major recovery over the past 15 years, with the government's economic recovery programme launched in 1983. Given the significant contributions identified, the paper concluded that the mining industry in Ghana is sustainable and the government is currently focusing on implementing these policy initiatives [8]. On the basis of analysing the characteristics of water use in various industries of the national economy, the author proposes a method to quantitatively determine a water-saving and high-efficiency water-use social production system, and establishes a water resource input-output analysis model, which will be applied to the actual situation in Beijing. Situation analysis [9]. The development of tourism plays an important role in adjusting the national economic structure and optimizing the enterprise structure. However, the status of tourism in the national economy is still a controversial topic, and the research results not only objectively reflect the status of tourism in the national economy but also improve the insufficiency of tourism statistics and industry contribution assessment [10]. The green economy is usually not a drag on growth, but a new engine of growth and an important strategy for eradicating persistent poverty. At the same time, there is growing evidence that the future is heading for a new economic paradigm—one in which the provision of material wealth is not necessarily accompanied by growing environmental risks, ecological scarcity, and social inequality at the expense [11]. The report gives a shocking figure, investing 2% of domestic GDP in 10 sectors of the green economy. This has important significance for social harmony and economic development, and green economy is a way to promote sustainable development at the global, national, and regional levels [12]. From local to global, scientists and communities must support systems for life on Earth and meet the needs of human development. This study shows that efforts to promote sustainable development are more likely to succeed if they are used to protect the boundary between knowledge and action while enhancing the visibility, credibility, and legitimacy of the knowledge they generate [13]. In this paper, we propose and rationally analyse the concept of the environment (EKC). It is considered that the relationship between environmental pollution and per capita income is inverted U-shaped, thus reducing the impact of economic activities on the environment, a concept based on an economic model in which environmental quality affects production opportunities and does not affect environmental degradation [14]. The past decade has seen a series of increasingly active movements using science and technology to seek the transition to sustainable development. These campaigns are based on broadness, that is, the challenge of sustainable development is to reconcile social development goals with the Earth's long-term environmental protection goals [15].

## 2. The Theoretical Framework of Sustainable Economic Development

### 2.1. The Concept of Sustainable Development

The concept of sustainable development shows that the carrying capacity of the environment and ecology is not infinite, and the total amount of natural resources is also limited. For a long time, only renewable resources can ensure the sustainability of development. The development process will only be sustainable if it is ensured that the overall capacity remains the same or increases over time. Sustainable development is a benign development process with an upward trend. This new development concept has three basic characteristics: First, sustainable development is balanced. Sustainable development emphasizes the balanced development of regions. Sustainable development requires each region to develop independently and not affect each other, that is, today's efforts are for a better tomorrow; the other is the harmonious development of man and nature in sustainable development. Sustainable circularity for continued development: sustainable development is a spiral development process. In such a vicious and virtuous cycle, it is necessary to select an appropriate development speed and scale according to the development capabilities such as resource capacity and environmental capacity.

### 2.2. Quantitative Measurement of Sustainable Development

Quantitative measurement of sustainable development is one of the core issues and theoretical frontiers of relevant economics research. Quantitative measurement of sustainable development mainly focuses on the sustainable development index system. The construction of the current international sustainable development indicator system and its calculation method generally conforms to two ideas: one is to incorporate sustainable development into the national accounts system, expand the current GDP and its system framework, and build an environmental and economic accounting system, including traditional economic accounts. The second is to follow the general idea of sustainable development theory and build a statistical index system and evaluation model reflecting sustainable development. There are two different opinions. One is to advocate the ability, performance, and achievement of sustainable development to be measured by a single comprehensive statistical indicator;

### 2.3. The Core of Sustainable Development Is Sustainable Economic Development

The core of sustainable development is sustainable economic development, while developed countries propose to focus on sustainable development of the environment, such as environmental pollution and nature protection. Therefore, their environmental protection concept is based on the relatively developed economy, and their understanding of the concept of sustainable development expresses their support for sustainability. Sustainable development can be understood as a dynamic process. In the short term, due to pressures such as “poverty,” economic development becomes a key theme, and as environmental conditions deteriorate, “environmental protection” becomes relatively important worldwide. Economic development requires the coordination of environment and development. Sustainable development has become an ideal model of economic development and an important part of sustainable economic development. It is also the sustainable growth of the economy and the profitability of people's production and business activities. With the continuous development of society, more and more attention has been paid to the stable and sustainable supply of natural resources and the environment, which is not only the premise of economic growth but also the premise of sustainable economic growth and coordination of resources and environment.

### 2.4. Analysis of Elements of Sustainable Economic Development

The debate on the factors of economic growth is not only a central issue in economics but also one of the longest and most debated topics in the history of economic thought. As economists struggle to explain the continued growth in people's productivity and incomes, they find that understanding this complex phenomenon requires adding more and more elements to the analytical framework.

In 1950, the economic circle put forward the total production function relationship that reflects the input of capital, labour, etc., and the expected return. So far, the theory that labour has a positive impact on economic growth has begun to revive. Some theories of the last century even believed that population growth was the main driving force of economic growth. Economists no longer look at economic growth from the perspective of a specific production function, recognizing that better technology can improve the level of the production function. Factors such as high savings rates, high levels of education, and positive technological innovation are signs of development associated with economic growth, facts explained by economic development theories, and not causes of development. We should also pay attention to the impact of natural resources and the environment on economic growth; especially since 1990, the concept of “sustainable development” was introduced in the analysis of sustainable economic long-term growth, and the incorporation of the environment into the analytical framework has become a solid economic an indispensable prerequisite for sustainable development theory (Figure 1).

China's extensive economic growth has come at the expense of environmental pollution. At present, China's economic growth is slow, and the problem of environmental pollution cannot be ignored. Empirical analysis shows that the overall model of economic growth at the expense of the environment is unsustainable; in other words, environmental inefficiency and unsustainable development hinder economic development and make sustainable economic development impossible; environmental protection efficiency and sustainable development are a prerequisite for achieving sustainable economic development.

## 3. Study on the Relationship between Economic Development and Ecological Environment Protection

### 3.1. Establish an Index System and Standardize It

#### 3.1.1. Index System Construction and Index Selection

The economy and environment are two very complex systems, and it is difficult to construct a relevant indicator system. Therefore, this paper is based on four principles: scientificity, accuracy, practicability, and unity. Based on the research experience of the researchers, and taking the regional economy as an example, an indicator system for the coordinated development of the regional economy and the ecological environment has been established.

#### 3.1.2. Standardization of Indicators

In the actual operation of the evaluation object with multiple attribute indicators, it is usually necessary to process the evaluation value of the standard evaluation object to eliminate the dimensional difference between various indicators, such as appropriate transformation of indicators of different sizes, removing the effects of nature, units, and quantities between individual data, and converting all data to the same size and into unmeasurable standardized indicators. We know that the economy and ecosystem are two very complex systems, and the relevant indicators are economy, society, resources, environment, etc., and must be analysed in multiple dimensions. If the collected data are directly applied to the relational calculation, there may be errors in the calculation results. The advantage of the range transformation method is that the index value satisfies 0 ≤ *y*_*ij*_ ≤ 1. Higher values of positive indicators indicate better economic and environmental performance, and there is a positive correlation between them and vice versa.

Suppose the eigenvectors of the environmental system and the economic system are $\bar{X_{ij}}=\left(X_{i1},X_{i2},X_{i3},\ldots ,X_{ij}\right)$; normalizing *X*_*ij*_ gets

(1) When *X*_*ij*_ is a positive correlation indicator:
  (1) $$\begin{array}{c} \bar{X_{ij}}=\frac{X_{ij}-X_{j\min}}{X_{j\max}-X_{j\min}}. \end{array}$$
(2) When *X*_*ij*_ is a negative correlation indicator:
  (2) $$\begin{array}{c} \bar{X_{ij}}=\frac{X_{j\max}-X_{ij}}{X_{j\max}-X_{j\min}}. \end{array}$$
Among them, *X*_*ij*_ represents the *i*-th actual observed value of the *j*-th indicator, *X*_*j*max_, *X*_*j*min_ represent the maximum and minimum values of the *j*-th indicator, and $\bar{X_{ij}}$ is the standardized data.

The indicator weight refers to the quantitative value of the proportion of each indicator of the measured object, which can also be called the sum of the weight factor and the indicator, and the indicators at each level should be weighted for calculation. The data are standardized to determine the entropy of the information. The data entropy of the *j* indicators can be defined as follows:

(3) $$\begin{array}{c} E_{j}=-\frac{1}{\ln\;m}\left(\sum_{i}^{m}F_{ij}\ln\;F_{ij}\right). \end{array}$$

In the formula, *F*_*ij*_ is the standardized value of the index data *X*_*ij*_. Finally, according to the formula to determine the index entropy weight *W*_*j*_, the formula is as follows:

(4) $$\begin{array}{c} W_{j}=\frac{1-E_{j}}{n-\sum_{j}^{n}E_{j}}, \end{array}$$

where *i* and *j* start from 1, *m* is the year, and *n* is the number of indicators. According to the above steps, the weights of the regional economic system and environmental system indicators are calculated as shown in Table 1.

### 3.2. Model Establishment

#### 3.2.1. Comprehensive Evaluation Model of Regional Economy

A comprehensive evaluation model of the regional economy is constructed, and the evaluation formula is as follows:

(5) $$\begin{array}{c} f\left(x\right)=\sum_{i=1}^{n}a_{i}x_{i}. \end{array}$$

Among them, *n* is the number of indicators, *a*_*i*_ is the indicator weight, and *x*_*i*_ is the standardized data.

#### 3.2.2. Regional Comprehensive Environmental Assessment Model

To construct a regional environmental comprehensive evaluation model, the evaluation formula is as follows:

(6) $$\begin{array}{c} g\left(y\right)=\sum_{i=1}^{m}b_{i}y_{i}. \end{array}$$

Among them, *m* represents the number of indicators, *b*_*i*_ represents the weight of the indicators, and *y*_*i*_ is the standardized data.

### 3.3. Regional Economy and Environment Coupling Degree and Coupling Coordination Degree Model

The degree of coupling is related to the degree of interaction between systems. It is used to measure the degree of granularity between systems and the relationship between different internal elements of the system. It can also measure the level of coordination between the economy and the environment in a country or region. The coefficient of variation is used to derive a computational model for the degree of coupling between the economy and the environment. When comparing the decomposition degrees of two data sets, if the number of the two data sets is too large or the comparison dimension is too large, the standard deviation should not be used. It just so happens that the coefficient of variation can replace the standard deviation method, measuring the variance, the higher the mean of the variable, the greater the dispersion, and vice versa. The formula for the coefficient of variation is as follows:

(7) $$\begin{array}{c} C_{v}=\frac{2S}{\left[f_{\left(x\right)}+g_{\left(y\right)}\right]}. \end{array}$$

Coefficient of variation: when the scatter of two data sequences needs to be compared, and the scale difference between the two data sequences is too large, the coefficient of variation can eliminate the influence of scale and measure, where *S* is the standard deviation. The formula for determining the degree of coordination between economy and environment is as follows:

(8) $$\begin{array}{c} c={\left\{\frac{f_{x}\times g_{y}}{{\left[\left(f_{x}+g_{y}\right)/2\right]}^{2}}\right\}}^{k}. \end{array}$$

Among them, *C*, *f*(*x*), and *g*(*y*) are the coupling degree, economic aggregate level, and environmental aggregate level, respectively, and *K* is the correction factor, which generally ranges from 2 to 5, and *K* is 4. The degree of coupling indicates that the level of coordinated development of the economy and the environment is positively correlated. The coupling model sometimes produces results that are inconsistent with the actual situation, and it is impossible to analyse whether the relationship between them is positive or negative. For example, the two regions have the same degree of connection between the environment and the economy, but it is possible that one region has a higher level of integrated development of the environment and the economy, while the other region is just the opposite, and its objective authenticity remains to be explored. The functional model of the coordination degree *D* is as follows:

(9) $$\begin{array}{c} D={\left(C\times T\right)}^{1/2},\\ T=\left(\alpha +\beta \right)\left(f_{y}+f_{x}\right). \end{array}$$

Among them, *D* is the coupling coordination degree, *T* is the overall economic and environmental development evaluation index, and *α* and *β* are the weights of each subsystem. Since the economic subsystem and ecological subsystem are of equal importance in the research process, the given value *α* = *β* = 0.5, and the value range of *D* is 0-1. This is the definition of the degree of interconnected coordination.

### 3.4. Forecast of Coordinated Development between Economic Development and Ecological Environment Protection

In order to better understand the constraints of regional economic and environmental development and the future development situation, to predict the degree of coordination between the regional economy and the environment, and the future economic and ecological conditions from 2007 to 2017, a GM (1, 1) model was constructed.

#### 3.4.1. Principle of GM (1.1)

Let *X*^(0)^ be the modelling sequence of GM (1, 1), *X*^(1)^ be the one-time accumulation sequence, and let *Z*^(1)^ be the generation sequence of the mean value (MEAN) of *X*^(1)^'s immediate neighbours, then the following relationship is obtained:

(10) $$\begin{array}{c} X^{0}=\left(x^{0}\left(1\right),x^{0}\left(2\right),\ldots ,x^{0}\left(n\right)\right),\\ X^{1}=\left(x^{0}\left(1\right),x^{1}\left(2\right),\ldots x^{0}\left(n\right)\right),\\ x^{1}\left(k\right)=\sum_{i=1}^{k}x^{0}\left(i\right),\;k=1,2,\ldots ,n,\\ Z^{1}\left(k\right)=\frac{1}{2}x^{1}\left(2k-1\right),\;k=2,3,\ldots ,n. \end{array}$$

Then, the definition type of GM (1, 1), that is, the grey differential equation model of GM (1, 1) is as follows:

(11) $$\begin{array}{c} x^{0}\left(k\right)+az\left(k+1\right)=b, \end{array}$$

where a is the development factor and *b* is the grey action. The bleaching equation (shading equation) of the grayscale differential equation is as follows:

(12) $$\begin{array}{c} \frac{\text{d}x^{2}}{d\left(t\right)}+ax=kb. \end{array}$$

As mentioned above, there is a solution to the whitening equation, also known as the time-response function, which is expressed as formula (13), and the time-response sequence of the GM (1, 1) grey differential equation is expressed as formula (14), and the reduction of the grey differential equation is further obtained. The value is shown in Equation (15).

(13) $$\begin{array}{c} x\left(t\right)=\left(ex-\frac{b}{a}\right)+\frac{b}{a}e^{at}, \end{array}$$

(14) $$\begin{array}{c} x\left(k+1\right)=\left[kx-\frac{b}{a}\right]e^{-ak}+\frac{b}{a}e^{ak}, \end{array}$$

(15) $$\begin{array}{c} x^{1}\left(k+1\right)=x^{0}\left(2k-1\right). \end{array}$$

#### 3.4.2. Model Establishment

According to the above GM (1, 1) principle, all *λ* are within the public coverage, so the original sequence does not need to be processed by the attenuation buffer operator, but a GM (1, 1) model can be established for it.

(16) $$\begin{array}{c} \lambda_{k}=\frac{x^{\left(0\right)}\left(k-1\right)}{x^{\left(0\right)}\left(k\right)},\;k=2,3,\ldots ,11. \end{array}$$

Construct an accumulation sequence once:

(17) $$\begin{array}{c} X^{\left(1\right)}=\left(x^{\left(0\right)}\left(1\right),x^{\left(0\right)}\left(2\right),\ldots x^{\left(0\right)}\left(n\right)\right)=\left(0.4290,0.9771,\ldots ,6.1376,6.9776\right). \end{array}$$

Finally, the prediction model is obtained:

(18) $$\begin{array}{c} \frac{\text{d}x^{\left(1\right)}}{\text{d}t}-0.0454x^{\left(1\right)}=0.4979, \end{array}$$

(19) $$\begin{array}{c} x^{\left(1\right)}\left(k+1\right)=\left[x^{\left(0\right)}\left(1\right)-\frac{b}{a}\right]e^{-ak}+\frac{b}{a}=11.3932e^{0.054k}-10.9642. \end{array}$$

To sum up, the established GM (1, 1) model is scientific. In this model, the data from 2018 to 2025 are first predicted; since the data collection will not end until 2025, the degree of linkage between the regional economy and the environment in 2018 and 2019 is predicted. The prediction results are shown in Table 2.

It can be seen from Table 2 that the coordination degree between regional economy and environment has improved from 2018 to 2025, and the development level of interconnection in the next 8 years has also changed from good coordination and optimization to quality coordination. This shows that the transformation and promotion of the regional economy, the support of relevant government policies, the continuous improvement of people's living standards, and the popularization of environmental protection concepts have all contributed to the coordinated development of the regional economy and environment, and are developing in a sustainable direction.

## 4. Empirical Research on Sustainable Development of Ecological Environment

### 4.1. Instance Selection

In recent years, Leshan's social economy has developed rapidly. The economic growth rate of Leshan has exceeded 10% in recent years. Leshan has become a world famous tourist city based on economic conditions alone. The environment has also changed dramatically. Therefore, we choose Leshan City as the representative to study the key factors of ecological environmental protection in sustainable economic development. The continuous expansion of urban buildings and public spaces, the continuous increase in the population base, the continuous increase in various industrial and domestic garbage dumps, and the decline in living comfort, traffic congestion, and noise pollution have caused serious impacts on the ecological environment and the sustainable development of urban areas, which seriously threatens the sustainable development goals of Leshan City. We have conducted a comprehensive study on the urban ecology and economic sustainability of Leshan, and put forward reasonable suggestions to improve the ecological sustainability of the urban environment. Promoting environmental harmony is of far-reaching significance and is conducive to the sustainable development of economy, society, and environment.

### 4.2. Calculation of Various Indices of Urban Ecological Environment

Using the calculation method of ecological indicators, refer to the “Leshan City Statistical Yearbook 2016–2020,” “Environmental Quality Report,” “City Quantitative Evaluation,” and other materials and obtain the relevant data of Leshan City from the four levels of different standards in the city (Table 3).

Engel coefficient is an important symbol to measure the wealth of a region or country. Generally speaking, under all conditions being equal, the higher the Engel coefficient, the lower the regional total profit and lower the gross national income, and vice versa. Table 3 shows that from 2016 to 2020, the social, economic, and natural environment of Leshan City underwent significant changes. The population has not changed much, which shows that Leshan City has well implemented the national population policy and the control measures are effective; the per capita GDP has increased year by year, and the economic environment is better than above; with the development of the social economy, the disposable income of urban residents has also increased. With the continuous improvement, people's quality of life has improved. At the same time, the Engel coefficient and the urban-rural income gap have narrowed; not only the living conditions of urban residents have been improved but the social and economic environment of the rural population has also been greatly improved. However, the urban-rural income gap still exists. To improve this situation, it is necessary to further increase rural incomes, improve the quality of life of farmers, and increase poverty alleviation projects, which must be based on effective government action.

As shown in Figure 2, from 2016 to 2020, the per capita public green space in Leshan City showed an increasing trend, but the trend was flat, and the per capita area was less than 22 square meters. But it also shows that from 2016 to 2020, the green area of Leshan City is on the rise, the green area has increased, and the environment has become more beautiful. The changes in per capita road area have different laws. Within 5 years, the per capita road area has increased, but the change has not changed much, indicating that the government does not pay enough attention to traffic roads.

At the same time, the 5-year GDP growth rate and Engel's coefficient (Figure 3) show that Leshan's economy and people's living standards have improved significantly over the past 5 years. By 2017, the GDP growth rate of Leshan City has exceeded 10%; especially in 2018, the growth rate was 18.7%, which was the year with the largest growth rate, but the economic growth rate will slow down in 2020. In recent years, the number of air pollution days has changed rapidly, and the number of air pollution days should increase slightly, indicating that environmental protection measures are still insufficient.

### 4.3. Analysis of Key Factors of Ecological Environment on Economic Development

As the economy develops, so does the quality of the natural environment (Figure 4). In 2020, the area of noise pollution in the whole district of Leshan City increased compared with 2016, decreased in 2018, and increased again in 2019. In 2017 and 2018, the area of water pollution increased compared with the previous year, and the remaining years decreased compared with the previous year. Especially in 2020, the area of water pollution fell to the lowest point in a year from 19 years. The occurrence of this situation is closely related to the environmental protection management measures in Leshan City. The increasing trend of water pollution areas in the past 2 years indicates that Leshan may have insufficient implementation of environmental protection measures, or pursue maximizing economic benefits while ignoring environmental impacts.

The organic whole of the social, economic, and natural environment forms the environment of the entire urban area. The three must develop in harmony in order to realize the protection of the ecological environment. Using the above estimation model, the secondary and primary index values of Leshan City were obtained according to Table 4 and Figure 5.

Figure 5 shows that from 2016 to 2020, the value of the secondary indicators of the social and economic environment in Leshan increased year by year. The growth rate was relatively stable in the first 2 years, but after 2018, the growth trend was obvious. It can be seen that the economic and social environment of Leshan City has improved significantly compared with previous years. In general, the social and economic environment of Leshan is getting better year by year. The difference is that the natural environment also showed an upward trend before 2017, but dropped sharply in 2018, indicating that the natural environment in Leshan in 2018 was worse than in previous years, but the natural environment in the following year improves.

However, as can be seen from Table 4, although the economic development has grown, the urban-rural income ratio is still relatively high. 2018 was the peak in the past 5 years. Since 2019, the urban-rural income ratio has declined, but the decline is small, indicating the urban-rural population. The income gap is still large; therefore, the urban sustainable development capacity can be divided into four levels according to the value of the urban ecosystem health index (Table 5).

According to Table 5, we can qualitatively evaluate the sustainable development of the ecological environment of Leshan City in the past 5 years (Table 6).

It can be seen from Tables 5 and 6 that the sustainability of the ecological environment in Leshan City is improving year by year. The improvement is not large enough, such as noise, water pollution, and air pollution days, and there is still room for improvement.

Figure 6 shows that from 2016 to 2020, the sustainable capacity of the ecological environment in Leshan City showed a steady growth trend, and the overall development trend was slow. In terms of comprehensive indicators, the environmental sustainability of Leshan has gradually increased from 0.541 in 2016 to 0.834 in 2020, which is mainly due to the rapid economic development of Leshan in recent years. According to the evaluation criteria of the index, the urban ecological environment of Leshan has developed from “moderate sustainable development, relatively harmonious economic environment and society” to the current level of “good sustainable development, harmonious economic environment and society.” Most of the indicators are moving towards excellent standards, indicating that the urban ecological environment of Leshan is gradually showing the harmonious development of society, economy, and nature.

### 4.4. Empirical Results

The main factors that promote the sustainable development of Leshan's ecological environment are the economic environment and the natural environment. The continuous improvement of Leshan's environmental remediation and environmental protection investment has significantly improved the overall quality of Leshan's urban environment, improved its pollution control capabilities, and achieved good results in ecological city construction. The main factor that promotes the sustainable development of Leshan's ecological environment is the social environment. The rapid economic development has brought enormous pressure to the urban environment. The construction of urban infrastructure is relatively lagging behind, which further affects the quality of life of residents. In addition, the energy consumption per 10,000 yuan of GDP is much higher than that of developed coastal cities, the unemployment rate remains high, and the water quality of major rivers is poor, which are important factors to promote the healthy and sustainable development of the regional economy.

## 5. Conclusions

From regional economic and environmental research to the sustainable development of the national economy, we find that the main factors that make positive contributions to the sustainable development of the ecological environment are the economic environment and the natural environment. Citizens' environmental awareness and environmental quality are sustainable, which are important part of development goals. To improve public awareness of environmental protection, it is necessary to improve residents' cultural literacy and ecological environment awareness through various means, so that all residents can consciously participate in urban ecological environmental protection activities and can pursue the concept of civilized ecological consumption in residents' lives. As far as the protection of the ecological environment is concerned, it is related to the sustainable and healthy development of the country's economy and society. “To promote its strengths and avoid its weaknesses,” on the basis of fully mobilizing the enthusiasm of the market economy participants, the ecological environment protection must be constantly reformed and improved. Measures, start from the particularity of the region and from the opposition and unity of economic development and environmental protection to find an effective way to solve the contradiction and finally achieve a benign interaction between the national ecological environment protection and economic development. The conceptual model of ecological footprint has been proposed for a short period of time, and there are not many cases of applied research in my country. There are still many areas for improvement in this model. From the specific situation of our country, it is necessary to do a good job in environmental protection to ensure sustainable development. Development research pushes to a higher analytical framework.

## Figures and Tables

**Figure 1:** Analysis of the elements of sustainable economic development.

**Figure 2:** Trend line of per capita public green space and road area.

**Figure 3:** Trend of economic index changes.

**Figure 4:** Changes in noise and water pollution areas.

**Figure 5:** Trend chart of secondary indicator values from 2016 to 2020.

**Figure 6:** Trend chart of sustainable development capability of ecological environment in Leshan City.

**Table 1:** Weights of regional economic and environmental system indicators.

Economic system	Weight	Environmental system	Weight
Total output value	0.165	Afforestation area	0.169
Total export-import volume	0.139	Land area covered with trees	0.152
Energy consumption per unit of GDP	0.153	Waste water discharge	0.155
Productivity of labour	0.158	Salvage value	0.148

**Table 2:** Predicted value of the coupling coordination degree between economy and environment in 2018–2025.

Year	Coupling coordination degree	Coupling coordination level
2018	0.8336	Good coordination
2019	0.8723	Good coordination
2020	0.9128	Quality coordination
2021	0.9552	Quality coordination
2022	0.9996	Quality coordination
2023	1.0406	Quality coordination
2024	1.0946	Quality coordination
2025	1.1455	Quality coordination

**Table 3:** 2016–2020 indicator data of Leshan City.

Name of index	2016	2017	2018	2019	2020
Density of population	0.0272	0.0271	0.0274	0.0273	0.0275
Per capita GDP	0.535	0.578	0.629	0.863	0.982
Per capita public green space area	15.24	16.43	17.68	19.91	21.67
Road area per capita	39.71	42.75	46.63	48.72	51.71
Engel coefficient (%)	37.2	36.5	35.2	34	33.1
GDP rate of rise (%)	9.5	18.2	18.7	17.6	14.1
Urban-rural income ratio	2.25	2.23	2.21	2.19	2.14

**Table 4:** Secondary index values in Leshan City.

Class	2016	2017	2018	2019	2020
Social environment	0.67	0.68	0.73	0.84	0.88
Economic environment	0.64	0.65	0.7	0.81	0.83
Natural environment	0.61	0.62	0.56	0.64	0.75

**Table 5:** The grading standard of urban ecological environment sustainability.

Grade	Exponential quantity	Qualitative evaluation
One	＞0.8	Fine
Two	0.6–0.8	Preferably
Three	0.4–0.6	Same as
Four	＜0.4	Very bad

**Table 6:** The first-level index values of Leshan City in 5 years.

	2016	2017	2018	2019	2020
Level 1 indicators	0.541	0.572	0.684	0.717	0.834
Qualitative evaluation	Same as	Same as	Preferably	Preferably	Fine

## Data Availability

The data used to support the findings of this study are available from the corresponding author upon request.
